The article "Clinical Effect of Side-Approach Laparoscopic Splenectomy for Neuropathic Splenomegaly" was retracted in 2023. Reasons: suspected computer-generated content; unreliable results or conclusions; lack of ethics approval or compliance; missing or withdrawn patient consent.

# Clinical Effect of Side-Approach Laparoscopic Splenectomy for Neuropathic Splenomegaly

**DOI:** 10.1155/2022/1224916

**Published:** 2022-05-09

**Authors:** Zhao Yuan, Hua Song An, Bo Yang, Hai Qing Li, Yuan Wang, Jian Wang

**Affiliations:** The Second Affiliated Hospital of Xuzhou Medical College, Hepatobiliary Pancreatic Surgery, 221000, China

## Abstract

**Objective:**

In order to investigate the clinical effect of side entry laparoscopic splenectomy in the treatment of splenomegaly caused by neurodegenerative diseases.

**Methods:**

62 patients who underwent endoscopic splenectomy in our hospital from July 2020 to June 2021 were randomly divided into two groups, including 3 cases in the observation group and 31 cases in the reference group. Clinical trials were conducted to compare different laparoscopic surgery methods, and follow-up investigation records were made; the drainage time and drainage volume, postoperative bleeding volume, postoperative complications, and comprehensive effective rate of the two groups were observed and analyzed.

**Results:**

Most of the drainage volume in the observation group was less than 800 ml, and most of the drainage volume in the reference group was more than 500 ml. Compared with the reference group, the average drainage time of patients in the observation group was lower, mostly within 6 days, while the drainage time of patients in the reference group was more than 8 days. The amount of bleeding in the observation group was mostly about 500 ml, with the largest number in the range of 300-500 ml, while the amount of bleeding in the reference group was mostly 800 ml and above, with the largest number in the range of 500-800 ml. The incidence of complications in the observation group was lower than that in the reference group. The effective, markedly effective and comprehensive effective rates of patients in the observation group were higher than those in the reference group, and the ineffective rate and deterioration rate were also lower.

**Conclusion:**

The treatment of lateral laparoscopic splenectomy is very safe and effective and has obvious advantages, because it can reduce the occurrence of postoperative complications and provide a good basis for the recovery of patients. It is worthy to be widely used in clinical splenic surgery.

## 1. Introduction

Splenomegaly is an important pathological feature, and the general causes are divided into infectious and noninfectious, and the texture of splenomegaly caused by different causes will change to different degrees. Splenectomy is often used as a treatment; this can correct the harm to the human body of splenomegaly, but the surgical resection of the whole spleen will also cause different degrees of immune function damage to patients. Because after total splenectomy, the filter plate function of the spleen will lead to disorders of the lymphatic system, with a significant decrease in lymphocyte number and conversion rate, which will increase the chance of fulminant infection and significantly increase [1].Compared with open splenectomy (OS), laparoscopic splenectomy (LS) can be applied in most diseases of the spleen requiring surgical resection; moreover, it has the advantages of minimally invasive surgery, such as small trauma, quick recovery, and short hospital stay [2].

Infectious patients are more prone to the spread of infectious lesions, while the main primary disease of noninfectious splenomegaly is leukemia, also known as malignant megalasplenia; at this time, the large incision operation is easy to cause the distant spread of malignant lesions. Therefore, radical splenomegaly is generally based on minimally invasive incision and endoscopy. Therefore, this study studies the clinical efficacy of different laparoscopic splenectomy in the treatment of splenomegaly.

## 2. Literature Review

Liu et al. compared the methods of splenectomy selected for different grades of splenomegaly. Open splenectomy can shorten the operation time and reduce the amount of intraoperative bleeding. It is safer to select OS than LS, especially for patients with grade IV splenomegaly [3]. Liu and Zhang showed that LS has the advantages of small surgical trauma, light pain, and fast recovery, and its safety and feasibility have been confirmed. However, the indications and contraindications of splenectomy should be strictly mastered in the later stage, and the appropriate operation should be selected for specific splenic diseases in order to achieve the best treatment [4]. Tang et al. studied the choice and clinical application value of laparoscopic splenectomy by secondary splenectomy and laparoscopic splenectomy by primary splenectomy, i.e., laparoscopic splenectomy by Endo-GIA division; after a retrospective analysis of the various patient results, it was found that laparoscopic splenectomy by secondary splenectomy has the advantages of low surgical cost and low complication rate; however, the operation process is relatively complex and requires high technical requirements for doctors, which requires rich experience [5]. Tang and Wan discussed the effect of “tunnel method” in the treatment of splenomegaly and believed that LS is safe and effective for conventional splenectomy or splenomegaly [6]. Gu discussed the safety and efficacy of LS in patients with hepatitis B cirrhosis after intravenous hypertension and splenomegaly. After analyzing 10 patients in the 105th Hospital of Chinese PLA, we concluded that LS is safe and effective in the treatment of patients with splenomegaly after portal hypertension [7]. Sheng et al. retrospectively analyzed the data of 55 cases of LS to explore the safety and efficacy of LS in various spleen diseases [8].

In the above literature review, all studies targeting splenomegaly therapy, but all of these studies are only the clinical studies of splenomegaly, the comparison of OS and LS, and the detailed studies in LS; there is no relevant research content for different LS. This study is conducted from this perspective; using the randomization method and using different LS for patients, the clinical efficacy of the patients of both groups was observed and analyzed; to find the best ways to reduce the surgical damage and bleeding and the occurrence of complications, efforts were made to improve the postoperative quality of life of the patients.

## 3. Data and Methods

### 3.1. General Information

62 patients who underwent endoscopic splenectomy from July 2020 to June 2021 were selected. All patients were diagnosed with infectious or malignant splenomegaly, excluding liver, lung, stomach, thoracic and abdominal nodules, tumors, and other space occupying lesions, and excluded diabetic patients. All patients were 22-56 years old, with an average age of 32.7 ± 5.5 years, the course of disease was 2-16 months, and the average course of disease was 4.3 ± 0.6 months. The difference in clinical general data of all patients was not statistically significant (*P* > 0.05).

The above patients were randomly divided into two groups, including 3 cases in the observation group and 31 cases in the reference group. After SPSS bivariate *t*-test analysis, the age, gender, course of disease, and other data of patients after grouping have *t* > 10.000 and *P* < 0.05, with credible statistical consistency. This clinical trial has been approved by the biomedical research ethics committee of Xuzhou Mining Group General Hospital with the approval number of (2019) 0020401.

### 3.2. Operation Method of the Observation Group

The patient was in the right decubitus position, inhalation general anesthesia, abduction fixation of the left upper limb, and headstock. During the operation, the bed structure adjustment and body structure pad height were used to adjust the body position. A 0.5-1.2 cm micro wound was cut in the left abdomen, and the carbon dioxide artificial pneumoperitoneum was 2 kPa. The first incision is 1.0 cm, located in the left quarter rib, between the umbilical and the left rib edge, as the endoscope inlet. The second incision is 1.2 cm, located in the posterior axillary line, between the iliac bone and the costal margin, as the main operation port. The third incision is 0.5 cm below the left costal margin and 10 cm away from the xiphoid process as an auxiliary operation port. If necessary, the main operation port can be expanded to 4.0 cm. After ligation of the main blood vessels of the spleen, a drainage tube was placed in the splenic fossa to prevent infection in the splenic fossa [9].

### 3.3. Operation Method of the Reference Group

The patient was in the right decubitus position, inhalation general anesthesia, abduction fixation of the left upper limb, and headstock. During the operation, the bed structure adjustment and body structure pad height were used to adjust the body position. A 0.5-1.2 cm micro wound was cut in the front abdomen and left abdomen, and carbon dioxide artificial pneumoperitoneum was 2 kPa. The first incision, 1.0 cm, is located in the periumbilical area as the endoscope inlet. The second incision, 1.2 cm, is located at the intersection of the left vertical line of the left central line of the left clavicle in the left middle and upper abdomen, and the third incision, 1.2 cm, is located at the projection area of the left anterior axillary axis through the splenic hilum for splenic ligament dissection and vascular ligation. The fourth and fifth incisions, 1.0 cm, are located at the connecting line between xiphoid process and navel for traction and fixation of the colon and stomach. If necessary, the main operation port can be expanded to 4.0 cm. After the main blood vessels of the spleen are ligated, the ligament tissue is stripped, cut, and taken out. Drainage tube was placed in splenic fossa.

### 3.4. Observation Contents and Diagnosis Methods

(1) Observe the indwelling time and drainage flow of the drainage tube in the splenic fossa, and the nursing staff or caregivers make statistics according to the recovery of the drainage bag
(2) The amount of postoperative bleeding, the number of bleeding cases, and their proportion were observed, and the statistics were made according to the clinical observation results during perioperative hospitalization and rehabilitation. If there is a need for supplementary surgery due to postoperative massive bleeding, the statistics were made according to the operation log data
(3) Observe the organic lesions and functional sequelae of the liver, gallbladder, stomach, colon, small intestine, peritoneum, and other organs of the thorax and abdomen within 6 months after operation. Those identified as medical accidents by the competent unit or appraisal institution shall be counted separately
(4) Observe the comprehensive effective rate of patients as follows:
  - *Remarkable Effect*. The patients had no significant postoperative complications and had high satisfaction with postoperative quality of life
  - *Effective*. The patients had no significant postoperative complications and the postoperative quality of life was basically satisfactory
  - *Ineffective*. The patient's discomfort caused by splenomegaly has not been improved, or there are postoperative complications
  - *Deterioration*. The patient has more serious complications after operation, or the primary symptoms worsen

### 3.5. Statistical Methods

The SPSS 22.0 statistical software was used for clinical data analysis, in which the counting data were used *χ*^2^. Conduct analysis and inspection and the measurement data adopts $\bar{x}\pm s$ indicate that bivariate *t*-test is used for continuous variable analysis. When *t* ≤ 10.000 and *P* < 0.05, it indicates that the data difference is statistically significant.

## 4. Results

### 4.1. Comparison of Postoperative Drainage Volume and Drainage Time

The drainage time and drainage volume of the two groups were statistically analyzed. The detailed data are shown in Tables 1 and 2.

In Table 1, most of the drainage volumes of patients in the observation group are distributed within 800 ml, and only a few are more than 800 ml, while most of the drainage volumes of patients in the reference group are distributed above 500 ml. All the statistical data have statistical differences. In order to more significantly compare the differences between the two groups, make a comparison according to Table 1 and as shown in Figure 1.

In Figure 1, it can be clearly seen that the distribution of drainage volume in the observation group is lower than that in the reference group, and there is only one observation group with drainage volume of more than 1200 ml, while there are three in the reference group, which shows that the drainage volume of patients treated with lateral laparoscopic splenectomy is much lower than that of patients treated with traditional laparoscopic splenectomy. This shows that the wound of side entry laparoscopic splenectomy is small, so the drainage volume is less.

In Table 2, it can be seen that there is a significant difference in the drainage time between the observation group and the reference group during the perioperative period (*P* < 0.05). Compared with the reference group, the average drainage time of patients in the observation group is lower, mostly within 6 days, while the drainage time of patients in the reference group is more than 8 days, in order to better observe the difference between the two groups of data, according to Table 2 and as shown in Figure 2.

In Figure 2, it can be clearly seen that the average drainage time of patients in the observation group is lower than that in the reference group, and there are 9 people in the observation group with drainage time less than 5 days, while there are only 3 people in the reference group, which shows that the recovery of side entry laparoscopic splenectomy is faster than that of traditional laparoscopic splenectomy.

### 4.2. Postoperative Bleeding Rate and Volume

The postoperative bleeding of patients will also reflect the operation and postoperative recovery. Therefore, the advantages and disadvantages of different laparoscopic splenectomy are analyzed by counting the bleeding volume and bleeding rate of the two groups. The detailed data are shown in Table 3.

In Table 3, according to the table data, the difference between the two groups is statistically significant (*P* < 0.05). It can be seen that the maximum amount of bleeding in the two groups is no more than 1500 ml, but the amount of bleeding in the observation group is mostly distributed around 500 ml, with the largest number in the range of 300-500 ml, while the amount of bleeding in the reference group is mostly 800 ml and above, with the largest number in the range of 500-800 ml. According to Table 3 and as shown in Figure 3, the difference between the two groups can be more clearly observed.

In Figure 3, it can be seen that the amount of postoperative bleeding of side entry laparoscopic splenectomy is significantly less than that of traditional laparoscopic splenectomy, because the wound of side entry laparoscopic splenectomy is small and the recovery is fast.

### 4.3. Postoperative Liver, Stomach, and Intestine Diseases

Patients after splenectomy may cause some complications, such as the liver, gallbladder, stomach, colon, small intestine, peritoneum, chest and abdominal cavity, and other organs. Therefore, the postoperative complications of the two groups within 6 months were investigated by follow-up [10]. The detailed data are shown in Table 4.

In Table 4, it can be seen that there is a statistical difference between the two groups (*P* < 0.05). Through the data comparison, the incidence of complications such as gastric disease, colon disease, small intestine disease, liver disease, and bile disease in the observation group is lower than that in the reference group. According to the data in Table 4 and Figure 4, the difference between the two groups of data can be more obvious.

In Figure 4, it can be seen that patients treated with lateral laparoscopic splenectomy have less postoperative complications. Therefore, this surgical method is recommended to reduce postoperative complications, improve the quality of life, and make patients recover faster and better.

### 4.4. Comprehensive Efficiency

Compare side entry laparoscopic splenectomy and traditional laparoscopic splenectomy, and select appropriate methods for patients. Compare the comprehensive effective rates of the two methods, in which the comprehensive effective rate = (markedly effective + effective)/2. The specific data are shown in Table 5.

In Table 5, it can be clearly seen that the effective, significant, and comprehensive effective rates of patients in the observation group are higher than those in the reference group, which shows that the effect of side entry laparoscopic splenectomy is better, and the ineffective rate and deterioration rate of patients in the observation group are also lower. In order to more clearly compare the differences between the two groups of data, make a comparative analysis as shown in Figure 5.

In Figure 5, it can be clearly seen from the histogram that the comprehensive effective rate of side entry laparoscopic splenectomy in the treatment of splenomegaly is high, which can effectively treat splenomegaly.

## 5. Discussion

Before the application of laparoscopic technology in clinic, OS is the only way for splenic surgery, but it has the disadvantages of large surgical wound, long postoperative recovery time, and many postoperative complications. The application of laparoscopic technology has opened the era of laparoscopic surgery and is a major change in the history of surgical hand. Li and Wang showed in the clinical application research of laparoscopic splenectomy that the continuous development of laparoscopic technology makes LS replace traditional OS as the preferred surgical method for splenectomy, and many types have been developed. Compared with OS, LS has the advantages of less trauma, rapid postoperative recovery, low incidence of complications, high safety, and good cosmetic effect, which is favored by doctors and patients [11]. Yu et al. showed that complete laparoscopic splenectomy via anterior approach is safe, feasible, and less invasive, which has obvious advantages over traditional laparoscopic splenectomy [12].

This study uses the method of clinical experiment to analyze the clinical effect of side entry laparoscopic splenectomy in the treatment of splenomegaly. Through the analysis of intraoperative drainage time, drainage volume, bleeding volume, and bleeding rate of patients in the two groups, it is found that when side entry laparoscopic splenectomy is used to treat splenomegaly, the drainage time is short, the drainage volume is less, and the postoperative bleeding volume is less. By means of follow-up, the postoperative complications of the two groups within 6 months were investigated, and the comprehensive effective rates of the two methods were compared. When lateral laparoscopic splenectomy was used to treat splenomegaly, the incidence of postoperative complications was small, and the comprehensive effective rate was high, which showed that the safety and curative effect of the operation were satisfactory.

## 6. Conclusion

In this study, the clinical effect of side entry laparoscopic splenectomy in the treatment of splenomegaly was analyzed by clinical experiment. Through the analysis of intraoperative drainage time and drainage volume in the two groups, it was found that the distribution of drainage volume in the observation group was lower than that in the reference group, and there was only one observation group with drainage volume of more than 1200 ml, while there were three in the reference group. This shows that the drainage volume of patients treated with side entry laparoscopic splenectomy is much lower than that of patients treated with traditional laparoscopic splenectomy, which shows that the wound of side entry laparoscopic splenectomy is small, so the drainage volume is less. By analyzing the amount of bleeding and bleeding rate of the two groups, it was found that the amount of postoperative bleeding of side entry laparoscopic splenectomy was significantly less than that of traditional laparoscopic splenectomy, because the wound of side entry laparoscopic splenectomy was small, and the recovery was fast. The postoperative complications of the two groups within 6 months were investigated by follow-up. It was found that the patients treated with lateral laparoscopic splenectomy had less postoperative complications. Therefore, this surgical method is recommended, which can reduce the postoperative complications, improve the quality of life, and make the patients recover faster and better. By comparing the comprehensive effective rates of the two methods, it is found that the effective, significant, and comprehensive effective rates of the patients in the observation group are higher than those in the reference group, which shows that the effect of side entry laparoscopic splenectomy is better, and the ineffective rate and deterioration rate of the patients in the observation group are also lower.

Therefore, for patients, the treatment of side entry laparoscopic splenectomy is very safe and effective, has obvious advantages, can reduce the occurrence of postoperative complications, and provides a good foundation for the recovery of patients. It is worthy to be widely used in clinical splenic surgery.

## Figures and Tables

**Figure 1:** Comparison of perioperative drainage volume between the observation group and the reference group.

**Figure 2:** Comparison of perioperative drainage time between the observation group and the reference group.

**Figure 3:** Comparison of postoperative bleeding between the observation group and the reference group.

**Figure 4:** Comparison of postoperative complications between the observation group and the reference group.

**Figure 5:** Comparison of comprehensive effective rate between the observation group and the reference group.

**Table 1:** Comparison of patients with different drainage volume between the two groups.

Grouping	Discharge				
	<300 ml	300-500 ml	500-800 ml	800-1200 ml	>1200 ml
Observation group	5	14	8	3	1
Reference group	1	8	10	9	3
*t*	7.264	7.354	7.138	7.601	7.806
*P*	0.031	0.037	0.035	0.032	0.046

**Table 2:** Comparison of the number of patients with different drainage time between the two groups.

Grouping	Drainage time				
	<5 d	5-6 d	6-8 d	8-10 d	>10 d
Observation group	9	11	6	3	2
Reference group	3	5	11	8	4
*t*	6.654	6.721	7.357	6.423	6.814
*P*	0.034	0.033	0.026	0.024	0.031

**Table 3:** Comparison of postoperative bleeding between the two groups.

Grouping	Bleeding volume				
	<300 ml	300-500 ml	500-800 ml	800-1500 ml	>1500 ml
Observation group	5	14	9	3	0
Reference group	2	6	15	6	2
*t*	5.364	5.213	5.621	5.372	5.206
*P*	0.026	0.024	0.021	0.031	0.034

**Table 4:** Incidence of complications within 6 months after operation in the two groups.

Grouping	Gastropathy	Colonic lesions	Small intestinal lesions	Liver lesion	Biliary lesions	Other lesions
Observation group	3	6	4	2	5	6
Reference group	7	11	8	9	13	14
*t*	3.254	3.314	3.322	3.214	3.621	3.312
*P*	0.036	0.039	0.041	0.038	0.046	0.042

**Table 5:** Comprehensive effective rate of the two groups.

Grouping	Remarkable effect %	Effective %	Invalid %	Deteriorate %	Comprehensive efficiency %
Observation group	94.24	96.18	7.35	3.54	95.21
Reference group	81.54	86.37	14.87	8.61	83.96
*t*	5.347	5.112	5.264	6.032	5.021
*P*	0.035	0.031	0.033	0.039	0.029

## Data Availability

The data underlying the results presented in the study are available within the manuscript.
